The article "A Physical-Chemical Study of the Interference of Ceftriaxone Antibiotic with Copper Chloride Salt" was published in 2021. Journal: Bioinorg Chem Appl.

# A Physical-Chemical Study of the Interference of Ceftriaxone Antibiotic with Copper Chloride Salt

**DOI:** 10.1155/2021/4018843

**Published:** 2021-10-19

**Authors:** Elsayed M. AbouElleef, Mowafak M. Mahrouka, Sherine E. Salem

**Affiliations:** ^1^Chemistry Department, Faculty of Arts and Science, Rafha Northern Border University, 91911 Rafha, Saudi Arabia; ^2^Basic Science Department, Delta Higher Institute for Engineering and Technology, Mansoura,, 35681 Dakhlia, Egypt; ^3^Chemistry Department, Faculty of Science, Mansoura University, 35516 Mansoura, Egypt

## Abstract

The nano-CuCl_2_.2H_2_O salt was prepared by the ball milling method. The association parameters for bulk and nano-CuCl_2_ salts in H_2_O are estimated at different temperatures using the conductivity method by applying the Fuoss–Shedlovsky equation and it was higher for nano-CuCl_2_ than bulk CuCl_2_ salt. The interaction between the cation (Cu^2+^) and ligand (ceftriaxone) in H_2_O was determined also by the conductometric method. Two stoichiometric complexes 1/2 and 1/1 (M/L) are estimated and follow the order *K*_f_ (1/1) > *K*_f_ (1 : 2) and ∆*G*_f_ (1/1) > ∆*G*_f_ (1/2) for (M : L) (in negative values) indicate the favorable of formation of (1/1) complex compared to the (1 : 2) complex. The Gibbs free energies change was increased in negative signs with increasing the temperature. The antimicrobial activities of CFT, bulk Cu-CFT complex, and nano-Cu-CFT complex were studied on LB agar by the disc diffusion technique against clinical isolates of gram-negative bacteria (*Klebsiella pneumonia* and *Pseudomonas aeruginosa*) and Fungi (*Candida albicans*). It was observed that (CFT) has a higher zone of inhibition and antibacterial activity than that of bulk and nano-Cu-CFT complexes in *Klebsiella pneumonia* and *Pseudomonas aeruginosa* (gram-negative bacteria). The nano-Cu-CFT complex showed a higher clear zone of inhibition and antifungal activity against candida than bulk Cu-CFT complex while the absence of the inhibition zone in CFT, so nano-Cu-CFT complex, can be used as an antifungal drug.

## 1. Introduction

Nanoparticles (NPs) are a wide class of materials that have a state between bulk and atomic or molecular structures in different shapes of 0D, 1D, 2D, or 3D and have a great scientific interest [1–5]. Bulk materials have constant physical properties, with size larger than one micrometer or micron. Nanoparticles can be used for various applications such as drug delivery purposes [6], diagnostics of cancer therapy, gene delivery purposes, chemical and biological sensing [7], gas sensing [8–10], CO_2_ capturing [11, 12], and other related applications [13–17]. Nanoparticles are often used to photocatalytically break down oil into biodegradable compounds, break down volatile organic pollutants in the air, and clean up carbon tetrachloride pollution in spring water [18, 19]. Nanoparticles (NPs) such as gold, silver, platinum, and palladium showed colors with the variation of shape and size and characteristic properties that can be utilized in bioimaging applications [20]. Another application of nanoparticles is the synthesis of photocatalysis S-doped TiO_2_ nanoparticles and the study of their photocatalytic, antimicrobial, and antioxidant activities under sunlight illumination [21].

Ceftriaxone [22–25] is an antibiotic that belongs to a category of medicine referred to as cephalosporin antibiotics, and it treats a variety of bacterial infections by stopping the growth of bacteria variety of bacterial infections (e.g., middle ear, lower tract, skin, and urinary tract), meningitis, gonorrhea, pelvic disease, and joint infections.

Thermodynamics parameters are an important tool for learning about the spontaneity of a given process at a particular temperature [26, 27]. Determination of the formation constant is fundamental for understanding the behavior of the metal cations in the presence of some chelating agent in a solution and is best explained using thermodynamics. A conductivity technique can be used to estimate the interaction between the metal cations and the chelating agent by estimating the thermodynamics parameters of metal-ligand complex formation [28–32].

It is therefore necessary to study the effect of antibiotic ceftriaxone on the properties of copper chloride salt by determining thermodynamics parameters of interaction between them using conductometric techniques to find the extent of benefit of the antibiotic ceftriaxone.

## 2. Experimental

### 2.1. Materials and Solutions

The purities and sources of the materials used are presented in Table 1. The structure of ceftriaxone is shown in Figure 1.

### 2.2. Apparatus

The conductance measurements are carried out with a conductometer A JENCO, Vision plus-EC3175 conductance instrument, and connecting with Kottermann ultra-thermostat-4130 (a deviation ±0.01 K) with a cell constant equal unity. The conductivity bridge was calibrated using standard potassium chloride solutions [33].

The Bruker *D*_8_ Advance X-ray diffractometer is a powder XRD instrument used to record X-ray diffraction (XRD) patterns of bulk and nanosamples. The Bruker diffractometer with CuK*α* anode radiation (*λ* = 0.1542 nm) as a source is operating at 40 kV and 30 mA. The scanning range of over an angular range was between 4° and 80°A at a temperature of 25°C, and the scan mode was applied with a step width of 0.02° per step and step time of 0.4 s.

IR instrument of the type Thermo Scientific Nicolet iS10 FTIR spectrometer is operating in the spectral range of 7800 to 400 cm^−1^ with a resolution of 4 cm^−1^, midinfrared KBr beamsplitter 4000 to 400 cm^−1^.

Solid samples can be prepared by grinding about 5 mg of sample mixed with 100 mg of spectroscopic grade KBr. This powder mixture is then compressed into a pellet using a mechanical press between 4 and 8 ton.cm^−2^ for 2 minutes in the form of 10 mm in diameter disks to form a translucent (http://en.wikipedia.org/wiki/Infrared_spectroscopy%20-%20cite_note-Har-2).

### 2.3. Procedure

#### 2.3.1. Preparation of Nanocopper Chloride

The nano-CuCl_2_.2H_2_O salt was prepared by the ball milling method by shaking CuCl_2_.2H_2_O salt in ball milling apparatus of the type Retsch MM 2000 swing mill at 20225 Hz at room temperature for one hour. The mill has 10 cm^3^ stainless steel double-walled tubes. Two balls made from stainless steel of 12 mm diameter were used.

#### 2.3.2. Preparation of Bulk Cu-CFT Complex and Nano-Cu-CFT Complex

Bulk Cu-CFT complex and nano-Cu-CFT were prepared according to a traditional method by refluxing 1 mmol of CFT under investigation with 1 mmol of bulk CuCl_2_.2H_2_O or nano-CuCl_2._2H_2_O salts in an ethanolic solution for 2-3 h close to the boiling point of the solvent. The precipitate was filtered off, washed several times with absolute ethanol, and finally dried in vacuum desiccators over anhydrous calcium chloride.

#### 2.3.3. Conductance Measurements

To calculate the association parameters of CuCl_2_.2H_2_O solutions, a solution of metal cation (10^−3^ M, 20 mL) was placed in a double jacket glass conductance cell, and the conductance was measured after each addition of the solvent and stirring at a specific temperature.

To calculate the formation constants between CuCl_2_.2H_2_O and a ligand (ceftriaxone) in the solvents, a solution of CuCl_2_.2H_2_O (10^−3^ M, 20 mL) was placed in a conductance cell, and the conductance was measured. The ligand (10^−3^ M) (ceftriaxone) was added step by step to the conductance cell using a micropipette and the conductance was measured after each addition.

#### 2.3.4. Biological Activity

The antimicrobial activities of CFT, bulk Cu-CFT complex, and nano-Cu-CFT complex were studied on LB agar by the disc diffusion technique against clinical isolates of gram-negative bacteria (*Klebsiella pneumonia* and *Pseudomonas aeruginosa)* and fungi (*Candida albicans*).

Sterile filter paper discs (6 mm) were individually immersed in dimethyl sulfoxide (DMSO) extract of CFT, bulk Cu-CFT complex, and nano-Cu-CFT complex, and DMSO was used as control. All the discs were dried, placed on the surface of the test bacterial and fungal, and incubated for 18 to 24 h at 37°C. The standard antibiotic used is ceftazidime (30 mg) and finally, the zones of inhibition were examined.

## 3. Results and Discussion

### 3.1. X-Ray Diffraction (XRD)

The X-ray diffraction (XRD) pattern for the bulk and nano-CuCl_2_.2H_2_O salt is shown in Figure 2. The positions of the main peaks and their relative intensities as measured by powder diffraction are listed in Table 2.

The mean size of nanocrystals was determined from the diffraction peaks corresponding to the most intensive reflections according to the Joint Committee on Powder Diffraction Standards database. Scherrer's equation was used to determine the average crystallite size for nanoparticles from the XRD diffraction pattern measured [34, 35]:

(1) $$\begin{array}{c} d=\frac{K\lambda }{\beta \;\cos\;\theta }, \end{array}$$

where *K* is Scherrer's constant (about 0.9), *λ* is the wavelength (*λ* = 0.154 nm), *β* is the line broadening at half the maximum intensity in radians, *θ* is the Bragg angle, and *d* is the averaged dimension of crystallites in nanometers. Groth assigned CuCl_2_·2H_2_O to the bipyramidal class of the orthorhombic crystalline system with the axial ratios *a* : *b* :  *c* = 0.9179 : 1: 0.4627. Layer line measurements give the identity distances *a*_0_ = 7.38 Å, *b*_0_ *=* 8.04 Å, *c*_*0*_ = 3.72 Å. These lead to the ratios *a* : *b* : *c* *=* 0.918 : 1: 0.462, in good agreement with the crystallographic data [36]. The mean crystal size (nm) of bulk and nano-CuCl_2_·2H_2_O salts obtained by XRD are mentioned in Table 2 [37].

A little difference was observed between bulk and nanosalts in peaks other than their intensities. Also, it was found that the salt remains in the crystalline form by converting it to nanoparticles. The main difference between the bulk and nanosalt was in the crystal size, as shown in Table 3.

### 3.2. Infrared Analysis (IR)

Infrared spectra (IR) were used to identify the structure of ceftriaxone (CFT), as shown in Figure 3, and its complexes with bulk and nano-CuCl_2_.2H_2_O salts as their functional groups give rise to characteristic bands in terms of both intensity and position (frequency), as shown in Figures 4 and 5.

It was observed from the IR spectra of ceftriaxone (CFT) ligand that amidic N-H stretching vibrations mean strong intensity bands occurring at 3440 and 3261 cm^−1^ are due to N-H asymmetric and symmetric stretching, respectively [38]. Amidic C=O stretching vibrations mean a strong intensity band identified at 1649 cm^−1^ is due to C=O stretching vibrations [38]. Amidic N-H deformation and C-N stretching mean the strong bands observed at 1608, 1537, and 1500 cm^−1^ are due to amide N-H deformation vibrations [38, 39]. C-H stretching vibrations mean the weak bands occurring at 2891 cm^−1^ are assigned to CH_3_ symmetric stretching. The bands appearing at 2934 cm^−1^ in the IR spectra are due to CH_3_ asymmetric stretching vibrations [40]. C-H deformation vibrations mean the weak bands observed at 822, 804, and 730 cm^−1^ are allotted as C-H out-of-plane deformation vibrations and medium-to-weak intensity bands present at 1104 and 1033 cm^−1^ are allotted as C-H in plane deformation vibrations. A strong band occurring at 1399 cm^−1^ is due to the -CH_2_- deformation vibration. Weak bands present at 1243 and 760 cm^−1^ are due to CH_2_ wagging and CH_2_ rocking vibrations, respectively [40]. Lactam C=O stretching vibrations mean a strong band observed at 1741 cm^−1^ in the IR spectrum of ceftriaxone is allotted to be due to C=O stretching vibration [41]. C-O-C stretching vibrations mean strong bands present at 1033 and 1243 cm^−1^ are assigned as C-O-C symmetric and asymmetric stretching vibrations, respectively [41]. C-S stretching vibrations mean weak bands observed at 646 and 616 cm^−1^ are due to C-S stretching vibrations [42]. C-N stretching vibrations mean the medium band present at 1285 cm^−1^, weak band at 1243 cm^−1^, and medium band present at 1185 cm^−1^ are due to C-N stretching vibrations. C=C and C=N stretching vibrations mean very strong intensity bands present at 1608, 1537, and 1500 cm^−1^ are assigned to C=C and C=N stretching vibrations [43]. O-H stretching vibrations mean strong intensity bands identified at 3440 and 3261 cm^−1^ are allotted as O-H stretching vibrations [44]. C-C and C-C-C bending vibrations mean a very weak band occurring at 507 cm^−1^ in is due to C-C out-of-plane bending vibrations. The weak bands occurring at 646 and 606 cm^−1^ are due to C-C-C in plane and out of plane deformation vibrations, respectively [45].

In the IR spectra of bulk Cu-CFT complex, as shown in Figure 4, after ceftriaxone coordination to copper ion, the frequencies of the (C=O) lactam shifted from 1741 cm^−1^ to higher wavenumber 1775 cm^−1^, one amidic (C=O) shifted from 1649 to lower wavenumber 1624 cm^−1^, and also another amidic (C=O) triazine shifted from 1608 to lower wavenumber 1553 cm^−1^. There are three functional groups participating in the formation of a complex. The increase in the vibrational frequencies of carbonyl groups can be explained by oxygen of lactam and triazine coordinating to Cu(II) indicates the formation of a chelate complex [46, 47]. These intramolecular interactions between oxygen and copper ion result in a more rigid molecular structure around the oxygen and shift of carbonyl (C=O) vibrational frequencies to higher wavenumbers. The frequency of the symmetric stretching mode *ν*_s_(COO−) shifts from 1391 to 1398 cm^−1^. These shifts indicate that the carboxylate group (COO), the lactam carbonyl group (C=O), and the oxo group of the triazine ring are involved in the formation of [Cu(CFT)]·3H_2_O. This analysis is in agreement with previous studies where ceftriaxone is described as a polydentate chelating ligand [46, 47]. The broadband in the [Cu(CFT)]·3H_2_O spectrum at 1624 cm^−1^ has a high intensity and a low resolution due to the overlap of several vibrational modes, including *ν*(C=O)-amide, *ν*(C=O)-triazine, *ν*_as_(COO–), *ν*(C=C), and *ν*(C=N). A new band appearing at the frequency 468 cm^−1^ in the complex that is absent in the free ligand is due to *ν* (Cu-N) stretching vibration also giving strong evidence for the coordination of tertiary nitrogen atom with copper ion [47].

Also, the IR spectra of nano-Cu-CFT complex asym.(NH_2_) shifted from 3440 to lower wavenumber 3427 cm^−1^, carboxylic (-OH) group appeared at wavenumber 2924 cm^−1^, carboxylic (C=O) appeared at wavenumber 1742 cm^−1^, one amidic (C=O) shifted from 1649 to lower wavenumber 1638 cm^−1^ and also another amidic (C=O) shifted from 1608 to lower wavenumber 1553 cm^−1^, as in Figure 5. This indicates the formation of a complex between CuCl_2_.2H_2_O salt and CFT antibiotic.

### 3.3. Conductometric Measurements

#### 3.3.1. Calculation of Association Parameters for Bulk and Nano-CuCl_2_·2H_2_O Salts in Distillate H_2_O

The specific conductance values (*K*_s_) of different concentrations of bulk and nano-CuCl_2_·2H_2_O salt in distillate H_2_O were measured experimentally in absence of (CFT) at different temperatures (288.15, 293.15, 298.15, and 303.15 K). The molar conductance (Λ_m_) values were calculated [48–50] using

(2) $$\begin{array}{c} \Lambda_{\text{m}}=\;\frac{\left(K_{s}-K_{\text{solv}}\right)\times 1000}{C}, \end{array}$$

where *K*_s_ and *K*_solv_ are the specific conductance of the solution and the solvent (distillate H_2_O), respectively, and C is the concentration of the bulk and nano-CuCl_2_·2H_2_O solutions.

The experimental data for conductance measurements were analyzed using Fuoss–Shedlovsky extrapolation techniques [51–53] which follow equations (3)–(12):

(3) $$\begin{array}{c} \frac{1}{\Lambda S_{\left(Z\right)}}=\frac{1}{\Lambda_{o}}+\left(\frac{K_{A}}{\Lambda_{o}^{2}}\right)\left(C\Lambda \gamma_{\pm }^{2}S_{\left(Z\right)}\right). \end{array}$$

The results obey the Fuoss–Shedlovsky equation and can be applied to obtain the value of limiting molar conductivity (Λ_o_) and association constant (*K*_A_) by plotting a graph between 1/Λ*S*(*z*) and (*C*Λ*S*(*z*)*γ*_±_^2^), which is presented in Figure 6, giving straight line with intercept (1/Λ_o_) and slope (*K*_A_/Λ_o_^2^):

(4) $$\begin{array}{c} S_{\left(Z\right)}=1+Z+\frac{Z^{2}}{2}+\frac{Z^{3}}{2}+\ldots , \end{array}$$

(5) $$\begin{array}{c} Z=\frac{S{\left(\Lambda C\right)}^{1/2}}{\Lambda_{0}^{3/2}}, \end{array}$$

(6) $$\begin{array}{c} S=a\Lambda_{0}+b, \end{array}$$

(7) $$\begin{array}{c} a=\frac{8.2\times 10^{5}}{{\left(\varepsilon T\right)}^{3/2}}, \end{array}$$

(8) $$\begin{array}{c} \left(\alpha \right)=\frac{\Lambda S_{\left(Z\right)}}{\Lambda_{0}}, \end{array}$$

(9) $$\begin{array}{c} \log\;\gamma_{\pm }=\frac{-A{\left(\alpha C\right)}^{1/2}}{\left[1+Br^{o}{\left(\alpha C\right)}^{1/2}\right]}, \end{array}$$

(10) $$\begin{array}{c} A=1.824\times 10^{6}{\left(\varepsilon T\right)}^{-3/2}, \end{array}$$

(11) $$\begin{array}{c} K_{A}=\frac{C_{\left[MX_{n}\right]}\cdot \gamma_{\left[MX_{n}\right]}}{C_{M^{n+}}\cdot \gamma_{M^{n+}}\cdot C_{X^{-}}^{n}\cdot \gamma_{X^{-}}^{n}}, \end{array}$$

where (*S*) is the Onsager slope; (*ε*) is the dielectric constant of the solvent,; (*η*_o_) is the viscosity of the solvent; (*T*) is the temperature; (*α*) is the degree of dissociation; (*γ*_±_) is the mean activity coefficients; (*z*^−^, *z*^+^) are the charges of ions in solutions; (*A*, *B*) are the Debye–Hückel constant; (*r*^o^) is the solvated radius; and (*K*_A_) is the association constant.

The dissociation constant (*K*_D_) is calculated by the following equation:

(12) $$\begin{array}{c} K_{D}=\frac{1}{K_{A}}. \end{array}$$

The Walden product (Λ_o_*η*_o_) values were calculated from the values of limiting molar conductance (Λ_o_) [54]:

(13) $$\begin{array}{c} \text{Walden product}=\Lambda_{o}\eta_{o}. \end{array}$$

The triple ion association constant *K*_3_ can be calculated from

(14) $$\begin{array}{c} \frac{\Lambda C^{1/2}}{{\left(1-\left(\Lambda /\Lambda_{o}\right)\right)}^{1/2}}=\frac{\Lambda_{o}}{{\left(K_{A}\right)}^{1/2}}+\frac{\lambda_{3}^{o}C}{K_{3}{\left(K_{A}\right)}^{1/2}}\left(1-\frac{\Lambda }{\Lambda_{o}}\right). \end{array}$$

The values of free energy of association (∆*G*_A_) of bulk and nano-CuCl_2_.2H_2_O salt in H_2_O at different temperatures of 288.15, 293.15, 298.15, and 303.15 K were calculated from the association constant *K*_A_ values [55] by using

(15) $$\begin{array}{c} \Delta G_{A}=-2.303RT\;\log\;K_{A}. \end{array}$$

The activation energy of the transfer process can be estimated depending on the relation between conductance of ion, ion mobility, and temperature degree, as in the Arrhenius equation:

(16) $$\begin{array}{c} \Lambda_{o}=Ae^{-E_{a}/RT}, \end{array}$$

where A is the frequency factor and *E*_a_ Arrhenius activation energy of the transport process.

(17) $$\begin{array}{c} \log\;\Lambda_{o}=\log\;Α-\frac{E_{a}}{2.303RT}. \end{array}$$

By plotting log Λ_o_ versus l/*T*, as shown in Figure 7, the activation energy of transfer processes values can be calculated from the slope [56].

The calculated values of Λ_o,_*S*_(*Z*)_, *α*, *γ*_±_, *K*_A_, *K*_D_, and *K*_3_ for the solutions of bulk and nano-CuCl_2_·2H_2_O salt with distillate H_2_O at different temperatures of 288.15, 293.15, 298.15, and 303.15 K are calculated and reported in Tables 4 and 5.

Table 4 shows that the limiting molar conductivity (Λ_o_) increases with increasing temperature due to the increase in mobility of ions and increasing kinetic energy which increases the separation among the oppositely charged ions while the Walden product (Λ_o_*η*) decreases with increasing the temperature due to the decrease in viscosity; also, the association constant (*K*_A_) decreases with increasing the temperature due to the decrease in the association of ions and the increase in mobility of ions; and similarly, the triple ion association constant (K_3_) decreases with increasing the temperature due to the decrease for the same reason.

Table 5 shows the same trend, that is, the limiting molar conductivity (Λ_o_) increases with increasing the temperature while the Walden product (Λ_o_*η*) decreases with increasing the temperature; also association constant (*K*_A_) decreases with increasing the temperature; and similarly, the triple ion association constant (*K*_3_) decreases with increasing the temperature.

The enthalpy (Δ*H*_*A*_) for bulk and nano-CuCl_2_·2H_2_O salts with distillate H_2_O at different temperatures were calculated by using Van 't Hoff equation:

(18) $$\begin{array}{c} \log\;K=-\frac{\Delta H}{2.303R}\left(\frac{1}{T}\right)+\text{constant}. \end{array}$$

By drawing the relation between log *K*_A_ and 1/T, Δ*H*_A_ can be calculated from the slope of each line which equals (-Δ*H*_A_/2.303 R), as shown in Figure 8. The entropy (Δ*S*_A_) for bulk and nano-CuCl_2_·2H_2_O salts were calculated by using

(19) $$\begin{array}{c} \Delta G_{A}=\Delta H_{A}-T\Delta S_{A}, \end{array}$$

where (*S*) is the entropy of the system. The calculated values of (Δ*H*_A_) and (Δ*S*_A_) for bulk and nano-CuCl_2_·2H_2_O salts are presented in Table 6. It is obvious that the limiting molar conductance (Λ_o_) increased as the temperature increased while the dissociation degree decreased as the temperature increased indicating a higher solvation process. The values of the association constant (*K*_A_) and the triple ion association constant (*K*_3_) were decreased by increasing the temperature. Gibbs free energies change of association (∆*G*_A_) was decreased with negative signs by increasing the temperature indicating that association is favored with lowering of dielectric constant of solvent mixture. The decrease in the values of activity coefficient, limiting molar conductance, association constant, Gibbs free energy change of association, and Walden product for nano-CuCl_2_·2H_2_O in comparison to bulk CuCl_2_·2H_2_O indicates that the association of nano-CuCl_2_·2H_2_O is greater than bulk CuCl_2_·2H_2_O salt, due to the high surface to volume ratio of nanoparticles which leads to a greater ability for ion-pair formation.

#### 3.3.2. Calculation of Formation Constants for Bulk and Nano-Cu-CFT Complexes in H_2_O at Different Temperatures

Different lines were obtained with breaks indicating the formation of (1 : 2) and (1 : 1) (*M* : *L*) stoichiometric complexes [57] on drawing the molar conductance (Λ_m_) for bulk and nano-Cu-CFT complexes at different temperatures versus the molar ratio of metal to ligand [*M*]/[*L*] concentrations, as shown in Figure 9.

The formation constants (*K*_f_) for bulk and nano-Cu-CFT complexes were calculated for each type of complexes (1 : 2) and (1 : 1) (M : L) by using

(20) $$\begin{array}{c} M^{2+}+L\;↔ML^{2+}, \end{array}$$

(21) $$\begin{array}{c} \left[L\right]={\left[L\right]}_{t}\;–\;\left\{{\left[M\right]}_{t}\frac{\Lambda_{M-\;}\Lambda_{\text{obs }}}{\left(\Lambda_{M-\;}\Lambda_{ML}\right)\;}\right\}, \end{array}$$

where Λ_m_ is the limiting molar conductance of the bulk and nano-CuCl_2_.2H_2_O alone, Λ_obs_ is the molar conductance of solution during titration, Λ_ML_ is the molar conductance of the complex, and [*L*] is the CFT concentration.

The Gibbs free energies changes of formation (Δ*G*_f_) for each stoichiometric complex were calculated [4] by using

(22) $$\begin{array}{c} \Delta G_{\text{f}}=-2.303RT\;\log\;K_{\text{f}}. \end{array}$$

The obtained values (*K*_f_) for bulk and nano-Cu-CFT complexes and their calculated Δ*G*_f_ values are presented in Tables 7 and 8.

By drawing the relation between log *K*_f_ and 1/*T*, different lines were obtained indicating the formation of (1 : 2) and (1 : 1) (*M* : *L*) stoichiometric complexes, as shown in Figure 10.

From the relation between log *K*_f_ and 1/*T*, Δ*H*_f_ can be calculated for each type of complexes, from the slope of each line which equals (−Δ*H*_f_/2.303 R). The entropy (Δ*S*_f_) for bulk and nano-Cu-CFT complexes was calculated for each type of complexes (1 : 2) and (1 : 1) (*M* : *L*) by using

(23) $$\begin{array}{c} \Delta G_{\text{f}}=\Delta H_{\text{f}}-T\Delta S_{\text{f}}. \end{array}$$

The calculated values of (Δ*H*_f_) and (Δ*S*_f_) for bulk and nano-Cu-CFT complexes are presented in Tables 9 and 10.

It was observed that inflections at (1 : 2) M/L proportion and (1 : 1) *M*/*L* indicating the formation of both stoichiometric complexes in the solutions. These types of stoichiometric complexes are formed as a result of the interaction of bulk or nano-CuCl_2_ with CFT in distillate H_2_O at different temperatures. The complex formation parameters for (1 : 1) complexes are greater than those of (1 : 2) complexes indicating more favorable complexes. Also, the complex formation parameters (*K*_f_, Δ*G*_f_) increased by increasing temperatures due to an increase in the kinetic energies. This trend was supported by entropies data which are greater for (1 : 1) *M*/*L* complexes than (1 : 2) *M*/*L* complexes.

## 4. Biological Activity

Many transition metals show arresting biological activity, working as active centers within important bioactive molecules in living systems. Copper (II) plays a significant function in cell metabolism and has proved beneficial in numerous diseases [58–60]. Ceftriaxone-metal complexes have both pharmacological and toxicological properties [61]. The interaction between metal ions and ceftriaxone can lead to precipitation resulting in serious adverse drug events [62]. Ceftriaxone complexes have antibacterial properties that can decrease or increase relative to pure ceftriaxone [61]. The antimicrobial activity was estimated based on the size of the inhibition zone formed around discs of bulk CuCl_2_·2H_2_O, nano-CuCl_2_·2H_2_O, CFT, and its bulk and nano-Cu complexes on a petri dish with Luria Bertani agar (LB-agar) plates as it measures the compound's efficacy.

### 4.1. Antibacterial Activity

The antibacterial activities of bulk CuCl_2_.2H_2_O, nano-CuCl_2_·2H_2_O, bulk and nano-Cu-CFT complexes were compared with the activity of CFT and as presented in Table 11. Bulk CuCl_2_·2H_2_O provides an excellent antimicrobial activity, and such property is greatly improved when using nano-CuCl_2_.2H_2_O. It was observed also that CFT has a higher zone of inhibition than bulk and nano-Cu-CFT complexes in *Klebsiella pneumonia* and *Pseudomonas aeruginosa* (gram-negative bacteria), Figure 11.

The antibacterial activity of Cu-CFT complexes depends on the bacterial species. The complexes and antibiotics presented inhibition zones of diameters larger than 20 mm showing that they have good activity as bactericides [63]. The antibacterial effect against *Staphylococcus aureus* is present at the bulk and nano-Cu-CFT complexes (the inhibition zones are 21 and 16 mm, respectively). These values are lower than the corresponding values for bulk CuCl_2_·2H_2_O and nano-CuCl_2_·2H_2_O and ceftriaxone. The data indicate that ceftriaxone ligand is more active than their metal complexes; this may be because the chelating ligands containing N and O donor atoms show wide biological activity through bonding to metal ions [64, 65]. However, the synergetic effects of ceftriaxone and Cu ion may play an important function in the inhibition of bacterial growth after the complex decomposition. These effects are due to the different mechanisms of the action of antibiotics and heavy ions on the bacteria metabolism [66, 67].

### 4.2. Antifungal Activity

The experimental antifungal activity data are presented in Table 11 which indicates that the nano-Cu-CFT complex showed a higher clear zone of inhibition against *Candida albicans* compared to the bulk Cu-CFT complex while there was an absence of the inhibition zone in CFT. So, the nano-Cu-CFT complex can be used as an antifungal drug, as shown in Figure 12. The zone of inhibition after treatment with bulk and nano-Cu-CFT complex was 8 and 9 mm, respectively. According to the standard criteria for evaluation of the drugs, the antifungal action such as a small zone of inhibition indicates that *Candida albicans* is stable with respect to CFT. The inhibition zones were completely absent, indicating the resistance of these fungi to CFT as well.

## 5. Conclusion

The nano-CuCl_2_·2H_2_O salt was prepared by ball milling method. The thermodynamic association parameters of both bulk and nano-CuCl_2_·2H_2_O salts in H_2_O were calculated using the conductometric method by applying the Fuoss–Shedlovsky method at different temperatures. It shows that the association parameters of nano-CuCl_2_·2H_2_O are greater than bulk CuCl_2_·2H_2_O salt due to the high surface-to-volume ratio of the nanoparticles which leads to a greater ability for ion-pair formation.

The thermodynamic parameters of complexation between bulk and nano-CuCl_2_·2H_2_O salts and ceftriaxone antibiotic in H_2_O were calculated from conductance measurement. It was found that the formation of Gibbs free energies change (∆*G*_f_) was decreased in negative signs with increasing temperatures. Two stoichiometric complexes, 1/2 and 1/1 (*M*/*L*), are formed with the formation constant and Gibbs free energy of the formed complexes following the order *K*_f_ (1 : 1) > *K*_f_ (1 : 2) for (M : L) and ∆*G*_f_ (1 : 1) > ∆*G*_f_ (1 : 2) for (*M* : *L*) (in negative values) indicates the favorable of formation of (1 : 1) complex compared to (1 : 2) complex. Also, there is a decrease in values of *K*_f_ and ∆*G*_f_ in case of using nano-CuCl_2_·2H_2_O compared to using bulk CuCl_2_·2H_2_O but in small difference due to the more solvation effect in case of using nanoparticles.

It was observed that CFT has a higher zone of inhibition and antibacterial activity than that of bulk and nano-Cu-CFT complexes in *Klebsiella pneumonia* and *Pseudomonas aeruginosa* (gram-negative bacteria). The nano-Cu-CFT complex showed a higher clear zone of inhibition and antifungal activity against *candida* compared to the bulk Cu-CFT complex while there was an absence of the inhibition zone in CFT, so the nano-Cu-CFT complex can be used as an antifungal drug.

## Figures and Tables

**Figure 1:** Molecular structure of ceftriaxone antibiotic (CFT). Formula: C_18_H_16_N_8_Na_2_O_7_S_3_.3.5H_2_O. Molar mass: 598.54 g/mol.

**Figure 2:** X-Ray diffraction of bulk and nano-CuCl_2_·2H_2_O salt.

**Figure 3:** IR spectra of ceftriaxone (CFT).

**Figure 4:** IR spectra of bulk Cu-CFT complex.

**Figure 5:** IR spectra of nano-Cu-CFT complex.

**Figure 6:** Variation of the molar conductance, l/Λ*S*_(*z*)_ with *C*Λ*γ*_±_^2^*S*_(*z*)_ for (a) bulk CuCl_2_·2H_2_O and (b) nano-CuCl_2_·2H_2_O in distillate H_2_O at (288.15, 293.15, 298.15, and 303.15) K.

**Figure 7:** Variation of log Λ_o_ with l/*T* (K^−1^) of for bulk and nano-CuCl_2_·2H_2_O in H_2_O.

**Figure 8:** Variation of log *K*_a_ with l/*T* (K^−1^) of for bulk and nano-CuCl_2_.2H_2_O in distillate H_2_O at 288.15, 293.15, 298.15, and 303.15 K.

**Figure 9:** The relation between Λ_m_ and the [M]/[L] molar ratio for (a) bulk Cu-CFT complex and (b) nano-Cu-CFT complex in distillate H_2_O at different temperatures.

**Figure 10:** Variation of log *K*_f_ with l/*T* for (a) bulk Cu-CFT complex and (b) nano-Cu-CFT complex in distillate H_2_O.

**Figure 11:** Inhibition zone around the discs (6 mm) containing (1) CFT, (2) bulk Cu-CFT complex, and (3) nano-Cu-CFT complex placed on the surface of an LB-agar plate with (a) *Klebsiella pneumonia* and (b) *Pseudomonas aeruginosa.*

**Figure 12:** Inhibition zone around the discs (6 mm) containing (1) CFT, (2) bulk Cu-CFT complex, and (3) nano-Cu-CFT complex placed on the surface of an LB-agar plate with *Candida albicans *.

**Table 1:** Sources and purity of the materials.

Chemical name	CAS reg. no.	Mass fraction	Purification method	Suppliers
Ceftriaxone	104376-79-6	0.990	Used as received	Sigma-Aldrich
Ethanol	64-17-5	0.995	Used as received	Sigma-Aldrich
CuCl_2_·2H_2_O	13464-92-1	0.980	Used as received	Sigma-Aldrich
H_2_O	7732-18-5	*k* < 0.5 *μ*S·cm^−1^	Distillation	Our lab
Mass fraction purity was provided by the suppliers.				

**Table 2:** Intensity (%) and crystal size (nm) of bulk and nano-CuCl_2_.2H_2_O salt.

Bulk CuCl_2_00B72H_2_O salt					Nano-CuCl_2_·2H_2_O salt				
Angle (2-theta °)	d value (angstrom)	Intensity (count)	Intensity %	Crystal size (nm)	Angle (2-theta °)	d value (angstrom)	Intensity (count)	Intensity %	Crystal size (nm)
16.375	5.40883	241	100	158.2	16.171	5.47654	28.5	76.8	16.171
22.097	4.01957	80	33.2	58.4	21.937	4.04841	20.4	55	21.937
26.76	3.32876	29.9	12.4	101.5	28.825	3.09476	24.5	65.9	28.825
28.938	3.08295	21.2	8.8	58.4	33.954	2.63814	37.1	100	33.954
32.916	2.71891	40.8	17	111.3	34.727	2.58114	13.3	35.9	34.727
35.491	2.52733	19.8	8.2	52.1	35.349	2.53715	13.3	35.8	35.349
38.19	2.35466	18.9	7.8	98.1	40.793	2.21025	17.2	46.3	40.793
44.933	2.01572	30.7	12.7	67.4	43.018	2.10094	11.2	30.1	43.018
49.254	1.84852	65.2	27.1	132.3	44.726	2.02457	13.3	35.9	44.726
50.199	1.81593	13.5	5.6	134.6	45.234	2.00303	13.6	36.5	45.234
54.558	1.68069	15.8	6.6	3	56.088	1.6384	10.8	29.1	56.088
57.572	1.59967	14.6	6.1	107.9	57.343	1.6055	16.1	43.4	57.343
63.915	1.45535	15.4	6.4	140.7	63.208	1.46991	9.72	26.2	63.208
68.788	1.36364	41.6	17.3						

**Table 3:** Mean crystal size (nm) of bulk and nano-CuCl_2_·2H_2_O salts.

Sample	Crystal size *d*_XRD_ (nm)
Bulk CuCl_2_.2H_2_O	94.146
Nano-CuCl_2_.2H_2_O	43.98

**Table 4:** Different association parameters (limiting molar conductance (Λ_o_), Fuoss–Shedlovsky parameter *S*_(*z*)_, degree of dissociation (*α*), activity coefficient (*γ*_±_), association constant (*K*_A_), dissociation constant (*K*_D_), triple ion association constant (*K*_3_)) for bulk CuCl_2_·2H_2_O in distillate H_2_O at 288.15, 293.15, 298.15, and 303.15 K in absence of CFT.

*T* (K)	Λ_o_*S*·cm^2^·mol^−1^	Λ_o_*η* S·cm^2^·MPa·s·mol^−1^	*α*	*γ*_±_	*K*_A_ dm^3^·mol^−1^	10^−3^*K*_D_ mol·dm^−3^	10^5^*K*_3_ (dm^3^·mol^−1^)^2^
288.15	270.00	307.43	0.9806	0.9022	99.74	0.0100	1.322
293.15	281.69	282.14	0.9668	0.9013	93.39	0.0107	1.273
298.15	284.90	254.16	0.9755	0.9005	82.79	0.0120	1.190
303.15	292.39	233.09	0.9912	0.8995	78.32	0.0127	1.154

**Table 5:** Different association parameters (limiting molar conductance (Λ_0_), Fuoss–Shedlovsky parameter *S*_(*z*)_, degree of dissociation (*α*), activity coefficient (*Ɣ*_±_), association constant (*K*_A_), dissociation constant (*K*_D_), triple ion association constant (*K*_3_)) for nano-CuCl_2_·2H_2_O in distillate H_2_O at 288.15, 293.15, 298.15, and 303.15 K in the absence of CFT.

*T* (K)	Λ_o_ S·cm^2^·mol^−1^	Λ_o_*η S*·cm^2^·MPa ·s·mol^−1^	*α*	*γ*_±_	*K*_A_ dm^3^·mol^−1^	10^−3^*K*_D_ mol dm^−3^	10^5^*K*_3_ (dm^3^·mol^−1^)^2^
288.15	266.21	302.58	0.9754	0.9022	60.60	0.0165	0.9949
293.15	271.73	282.14	0.9013	0.9013	56.35	0.0177	0.9546
298.15	277.00	247.11	0.9873	0.9005	46.16	0.0216	0.8499
303.15	282.48	225.19	0.9874	0.8995	34.47	0.0290	0.0714

**Table 6:** Gibbs free energy of association (Δ*G*_A_), enthalpy change (Δ*H*_A_), and entropy change (Δ*S*_A_) for bulk and nano-CuCl_2_·2H_2_O in distillate H_2_O at different temperatures.

T (K)	Δ*G*_A_ (kJ mol^−1^)		Δ*H*_A_ (kJ mol^−1^)		*E*_A_ (kJ mol^−1^)		Δ*S*_A_ (kJ mol^−1^K^−1^)	
	Bulk	Nano	Bulk	Nano	Bulk	Nano	Bulk	Nano
288.15	−11.028	−9.322					−0.0496	−0.0904
293.15	−11.059	−9.828	−12.928	−22.918	3.60	3.72	−0.0487	−0.0842
298.15	−10.949	−9.501					−0.0477	−0.0824
303.15	−10.993	−8.924					−0.0468	−0.0807

**Table 7:** Limiting molar conductance (Λ_o_) and formation constant (*K*_f_) for bulk Cu-CFT complex in distillate H_2_O at different temperatures.

*T* (K)	[*M*] : [*L*]	Λ_o_*S* cm^2^·mol^−1^	Λ_obs_*S* cm^2^·mol^−1^	log *K*_f_ dm^3^·mol^−1^
288.15	1 : 2	912.11	433.62	4.211
	1 : 1	554.03	440.05	4.424
293.15	1 : 2	958.50	473.22	4.186
	1 : 1	584.60	331.16	4.375
298.15	1 : 2	966.40	465.30	4.179
	1 : 1	594.50	322.25	4.342
303.15	1 : 2	985.30	481.14	4.174
	1 : 1	593.40	347.49	4.275

**Table 8:** Limiting molar conductance (Λ_o_) and formation constant (*K*_f_) for nano-Cu-CFT complex in distillate H_2_O at different temperatures.

*T* (K)	[*M*] : [*L*]	Λ_o_*S* cm^2^·mol^−1^	Λ_obs_*S* cm^2^·mol^−1^	Log *K*_f_ dm^3^·mol^−1^
288.15	1 : 2	912.00	439.56	4.191
	1 : 1	555.00	290.00	4.426
293.15	1 : 2	966.00	473.22	4.177
	1 : 1	593.00	331.16	4.349
298.15	1 : 2	958.00	485.10	4.180
	1 : 1	584.00	335.61	4.323
303.15	1 : 2	985.30	481.14	4.171
	1 : 1	593.00	348.98	4.263

**Table 9:** Different formation parameters (Gibbs free energy of formation (Δ*G*_f_), enthalpy change (Δ*H*_f_), and entropy change (Δ*S*_f_)) for bulk Cu-CFT complex in distillate H_2_O at different temperatures.

*T* (K)	Complex ratio (*M* : *L*)	Δ*G*_f_ (kJ mol^−1^)	Δ*H*_f_ (kJ mol^−1^)	Δ*S*_f_ (kJ mol^−1^K^−1^)
288.15	(1 : 2)	−23.23	−3.97	0.0252
293.15		−23.50		0.0257
298.15		−23.86		0.0265
303.15		−24.23		0.0273
288.15	(1 : 1)	−24.41	−15.96	0.0847
293.15		−24.56		0.0838
298.15		−24.79		0.0831
303.15		−24.82		0.0819

**Table 10:** Different formation parameters (Gibbs free energy of formation (Δ*G*_f_), enthalpy change (Δ*H*_f_), and entropy change (Δ*S*_f_)) for nano-Cu-CFT complex in distillate H_2_O at different temperatures.

*T* (K)	Complex ratio (*M* : *L*)	Δ*G*_f_ (kJ mol^−1^)	Δ*H*_f_ (kJ mol^−1^)	Δ*S*_f_ (kJ mol^−1^K^−1^)
288.15	(1 : 2)	−23.12	−1.82	0.0208
293.15		−23.44		0.0215
298.15		−23.86		0.0226
303.15		−24.21		0.0234
288.15	(1 : 1)	−24.42	−17.13	0.0847
293.15		−24.41		0.0833
298.15		24.68		0.0828
303.15		−24.75		0.0816

**Table 11:** Inhibition zones for antibacterial activity (gram-negative bacteria) and antifungal activity (*Candida albicans*).

Compound	Inhibition zone (mm)		
	Types of gram-negative bacteria		Type of fungi
	*Klebsiella pneumonia*	*Staphylococcus aureus*	*Candida albicans*
Bulk CuCl_2_·2H_2_O	19	17	12
Nano-CuCl_2_·2H_2_O	23	22	14
Ceftriaxone (CFT)	34	33	0
Bulk Cu-CFT complex	24	21	8
Nano-Cu-CFT complex	25	16	9

## Data Availability

The data are available on request from the corresponding author.
